This article has been retracted.

# Small Protein-Mediated Quorum Sensing in a Gram-Negative Bacterium

**DOI:** 10.1371/journal.pone.0029192

**Published:** 2011-12-12

**Authors:** Sang-Wook Han, Malinee Sriariyanun, Sang-Won Lee, Manoj Sharma, Ofir Bahar, Zachary Bower, Pamela C. Ronald

**Affiliations:** 1 Department of Plant Pathology and the Genome Center, University of California Davis, Davis, California, United States of America; 2 The Department of Plant Molecular System Biotechnology and Crop Biotech Institute, Kyung Hee University, Yongin, South Korea; Indian Institute of Science, India

## Abstract

The rice XA21 pattern recognition receptor binds a type I secreted sulfated peptide, called axY^S^22, derived from the Ax21 (activator of XA21-mediated immunity) protein. The conservation of Ax21 in all sequenced *Xanthomonas spp.* and closely related genera suggests that Ax21 serves a key biological function. Here we show that the predicted N-terminal sequence of Ax21 is cleaved prior to secretion outside the cell and that mature Ax21 serves as a quorum sensing (QS) factor in *Xanthomonas oryzae* pv. *oryzae*. Ax21-mediated QS controls motility, biofilm formation and virulence. We provide genetic evidence that the *Xoo* RaxH histidine kinase serves as the bacterial receptor for Ax21. This work establishes a critical role for small protein-mediated QS in a Gram-negative bacterium.

## Introduction

Given the demonstrated importance of plant and animal receptors [also called pattern recognition receptors (PRRs)] of conserved microbial signatures [also called pathogen associated molecular patterns (PAMPs)], there is great interest in elucidating the biological function of these ligands [1]. We have recently shown that the rice XA21 receptor binds a sulfated peptide, called axY^S^22, derived from the Ax21 (activator of XA21-mediated immunity) protein from the Gram-negative bacterium, *Xanthomonas oryzae* pv. *oryzae* (*Xoo)*. XA21/axY^S^22 binding triggers XA21-mediated innate immunity [2], [3].

The conservation of Ax21 in all sequenced *Xanthomonas spp., Xylella fastidiosa* and the human pathogen *Stenotrophomonas maltophilia* suggests that Ax21 serves a key biological function. To elucidate this function, we previously isolated and characterized eight genes required for Ax21 activity (*rax* genes). *raxA*, *raxB* and *raxC* encode components of a predicted type I secretion system (TOSS). Ax21 requires this RaxABC TOSS for activity and secretion [3], [4]. The RaxB protein carries two highly conserved N terminal proteolytic subdomains characteristic of transporters in Gram-positive bacteria that cleave N-terminal peptides prior to substrate secretion [4]. These data, together with the presence of a predicted N-terminal signal sequence in Ax21, suggest that Ax21 is cleaved by the RaxB transporter prior to secretion. *raxST*, *raxP* and *raxQ* encode enzymes involved in sulfation; and *raxH* and *raxR* encode a predicted histidine kinase and cognate response regulator, respectively [4], [5], [6]. The expression of the eight *rax* genes is density-dependent [7]. Their expression at low densities can be rescued by the addition of high-performance liquid chromatography (HPLC)-fractionated *Xoo* PXO99 supernatants. Fractions from *Xoo* strains lacking Ax21 activity cannot induce density dependent expression. We therefore, hypothesized that Ax21 serves as a quorum sensing (QS) factor.

QS is a process where small molecules serve as signals to recognize cell population size, leading to changes in expression of specific genes when the QS factor has accumulated to a certain threshold concentration [8]. In Gram-positive bacteria, QS is controlled by oligopeptides, whereas Gram-negative bacteria generally use acylated homoserine lactones (AHLs) or diffusible signal factors (DSF) for QS [9]. One instance of peptide-mediated QS in Gram-negative bacteria has been reported [10]. Although QS factors are abundant in the host vicinity, none have previously been shown to bind host receptors of conserved microbial signatures.

## Results and Discussion

To determine if Ax21 can serve as a QS factor to regulate density-dependent expression of *rax* genes, we monitored *rax* gene expression in PXO99 and in a mutant strain lacking Ax21 (PXO99*Δax21*). We found that the six *rax* genes were highly expressed in PXO99 cultures grown to high population densities [10^8^ colony forming unit (CFU)/ml], but not in PXO99*Δax21* cultures (Table. S1). These experiments indicate that Ax21 regulates density-dependent expression of *rax* genes.

We next purified Ax21 using gel filtration and immobilized metal ion affinity chromatography from culture supernatants of an *Xoo* strain expressing biologically active mature 6x-His-tagged Ax21 (rAx21) (without the N-terminal signal sequence) (Figure S1 and S2). A 7 kDa cut-off spin column was used to remove small peptides and other small molecules from the supernatants (Figure S2A). Elution was carried out using elution buffers containing various concentrations of imidazole (Figure S2B). Western blot analysis using an anti-Ax21 antibody revealed that the 150 mM imidazole buffer-eluted fraction contains highly purified rAX21 (Figure S2B).

To test whether the mature Ax21 protein itself could restore *rax* gene expression to the PXO99Δ*ax21* strain, we added rAx21 to this strain. We found that addition of the 150 mM imidazole-eluted fraction carrying rAx21, complemented *rax* gene expression in PXO99Δ*ax21* whereas addition of flow-through or 250 mM imidazole buffer-eluted fractions lacking rAx21 did not (Figure 1). Furthermore, the peptides, axY^S^22 and axM178, derived from Ax21 that were previously identified in HPLC-fractionated *Xoo* PXO99 supernatants [3], did not restore *rax* gene expression to the PXO99Δ*ax21* strain (Figure S4 and S5). These results conclusively demonstrate that the mature rAx21 protein serves as the QS factor and that the activity is not due to small peptides or other molecules present in the active fraction.

**Figure 1:** Purified recombinant Ax21 complements density-dependent expression of *raxST, raxB*, and *raxR* in PXO99*Δax21.* Expression of the *raxST, raxB,* and *raxR* genes in PXO99 (10^6^ and 10^8^ CFU/ml, grey), PXO99*Δax21* (10^8^ CFU/ml, black), and PXO99*Δax21* (10^8^ CFU/ml) supplemented with exogenous addition of the flow-through (FT), 150 mM (150), or 250 mM (250) imidazole buffer-eluted fractions (figure S2) was assessed. Levels of gene expression were calculated relative to 16sRNA expression. Primers specific to each gene are as listed in table S8. Data are mean of four replicates ± standard deviation (SD.).

As an additional test to investigate the nature of Ax21, we carried out liquid chromatography–tandem mass spectrometry of supernatants from PXO99Δ*ax21*(rAx21). Nine peptides spanning nearly entire Ax21 protein, except for the predicted N-terminal signal sequence were identified. These results demonstrate that the entire, mature Ax21 protein is secreted and that the predicted N-terminal signal sequence is cleaved before secretion (Figure S3).

To test if the biological activity of rAx21 is dependent on the predicted tyrosine sulfotransferase, RaxST, we isolated rAx21 from the PXO99Δr*axST* strain [4] expressing rAx21. rAx21 purified from this strain, displayed significantly less activity compared with rAx21 purified from the PXO99Δ*ax21* strain (Figure S6). These results indicate that RaxST is required for full Ax21 biological activity.

Bacteria use QS communication to regulate diverse biological processes, including motility, virulence and transition from a planktonic (free swimming) state to a sessile state, called a biofilm. To elucidate the biological function of Ax21, we compared expression profiles of PXO99 and PXO99*Δax21* at three different population densities. PXO99 and PXO99*Δax21* were diluted to 10^5^ CFU/ml and continuously grown until population densities reached 10^6^, 10^7^ and 10^8^ CFU/ml (representing early log, middle log, and late log phases of bacterial growth, respectively). RNA was then isolated and subjected to whole genome expression profiling. We found that 489 genes (approximately 10% of *Xoo* genome) are significantly differentially regulated by Ax21 (Figures S7, S8, S9 and Tables S1, S2, S3, S4, S5, S6, S7).

Ten of these genes encode proteins containing the amino acid domains GGDEF, EAL, and HD-GYP (Figure 2A). Such proteins have previously been shown to control cyclic diguanylate (c-di-GMP) turnover, a nucleotide-based secondary messenger that regulates diverse microbial phenotypes including growth, motility, virulence, and biofilm formation. In *Xanthomonas spp.,* the RpfC/G sensor kinase and response regulator are required for DSF perception and signal transduction leading to c-di-GMP degradation through a protein containing an HD-GYP domain [11]. In the opportunistic pathogen *Pseudomonas aeruginosa,* AHL-mediated c-di-GMP production is regulated by a tyrosine phosphatase (TpbA) [12]. Thus, three distinct QS systems (AHL-, DSF- and Ax21-mediated) control expression of genes encoding proteins that regulate c-di-GMP turnover. Bacterial c-di-GMP has also recently been shown to trigger the innate immune response of mouse and human cells [13], [14].

**Figure 2:** Whole genome transcriptomics of PXO99 vs. PXO99*Δax21* at different population densities identifies Ax21-regulated genes. A heat map represents the ratio of gene expression levels in a log_2_-based pseudocolor scale (red, positive; green, negative). (A) Expression pattern of genes encoding proteins predicted to regulate c-di-GMP turnover in PXO99 (Left) and PXO99*Δax21* (Right). (B) Ax21 up-regulated genes that are highly expressed in early log phase including bacterial motility genes and xanthan gum biosynthesis. The functions of the genes marked by a star were assessed for phenotypes in *Xoo* knockout strains (Figure S13).

Our expression analysis also identified a set of genes that are up-regulated by Ax21 during early log phase (Figure 2B). These include the *gumE*, *gumJ*, and *gumK* genes, which encode proteins required for biosynthesis of xanthan gum, an important component of the *Xanthomonas* extracellular polymeric substance (EPS) [15] (up-regulated by Ax21 2.0, 1.8, and 1.8 fold, respectively in PXO99 vs. PXO99Δ*ax21*). EPS enables bacteria to adhere to each other or to a solid surface, a key component of biofilms.

To assess if Ax21 is required for biofilm formation, we examined biofilm formation in the PXO99, PXO99Δ*ax21*, and PXO99Δ*raxST* strains using a plate adherence assay. The PXO99Δ*ax21* strain formed significantly less biofilms as compared with the PXO99 strain. Exogenous addition of purified rAx21 restored biofilm formation in PXO99Δ*ax21* (Figure 3A). Aggregation assays comparing PXO99Δ*ax21* and PXO99 revealed that Ax21 is also required for *in vivo* aggregation of *Xoo* (Figure 3B). Similar results were obtained using confocal microscopy (Figure S10). These experiments demonstrate that Ax21-mediated QS controls biofilm formation in *Xoo*.

**Figure 3:** Ax21 regulates *Xoo* biofilm formation, cell aggregation, motility, and virulence. (A) Biofilm formation of PXO99, PXO99*Δax21*, PXO99*Δax21* supplemented with exogenous addition of the flow-through (FT), 150 mM (150), or 250 mM (250) imidazole buffer-eluted fractions (figure S2) were measured according to absorbance at A_590_ using the polyvinyl chloride plate assay and normalized with the value of PXO99. Bars represent the mean of ten biological replicates ± SD. (B) Aggregation assays were performed using PXO99 and PXO99Δ*ax21* strains carrying a green fluorescent protein. *Xoo* strains were observed with a microscope equipped with a fluorescein isothiocyanate filter (excitation filter, 450 to 490 nm; emission filter, 520 nm; dichroic mirror, 510 nm). The bars indicate 10 µm. (C) Swimming motility of PXO99 and PXO99*Δax21* strains were quantified by measuring the diameter of colony expansion in swimming motility assays. Bars represent the mean of four biological replicates ± SD. (D) Virulence of PXO99 and PXO99*Δax21* was monitored at low population densities. Rice leaves (TP309 cultivar) were inoculated with PXO99, PXO99Δ*raxST*, and PXO99Δ*ax21* strains using the soaking method (10^3^ CFU/ml) for two days. Bacterial populations were determined two days after inoculation. Bars represent the mean from at least seven leaves ± SD. The experiment was repeated four times with similar results.

Our microarray data also revealed that, at early log phase, Ax21 up-regulates expression of genes involved in bacterial motility (Figure 2B). For example, *fliC*, *fliD* (flagella biosynthesis genes C and D) and the chemotaxis gene PXO_04752, are up-regulated 3.3-, 3.3-, and 16.4- fold, respectively in the PXO99 vs. PXO99Δ*ax21* strains. To test whether Ax21 controls *Xoo* motility, we assayed the phenotype of *Xoo* PXO99 and PXO99Δ*ax21* strains using a swimming motility plate assay. We found that the motility of PXO99 was two-fold higher than that of PXO99Δ*ax21* (Figure 3C) indicating that Ax21 regulates *Xoo* swimming motility on semi-solid media.

We have previously shown that the predicted histidine kinases PhoQ and RaxH are required for Ax21-mediated activities [5], [16]. We therefore hypothesized that one of these proteins was the bacterial receptor for Ax21. In support of this hypothesis, we observed that biofilm formation in both the PXO99*ΔraxH* and PXO99*ΔphoQ* strains is reduced compared to the PXO99 strain (Figure S11). We next tested whether biofilm activity could be rescued by addition of purified rAx21 protein to these mutant strains. We found that PXO99*ΔphoQ* but not PXO99*ΔraxH* could form biofilms after complementation with rAx21 (Figure S11). These results indicate that the defect in biofilm formation in PXO99*ΔphoQ* is not due to perception of Ax21. In contrast, the *Xoo* strain carrying a mutation in *raxH* could no longer respond to rAx21, supporting the hypothesis that RaxH is the Ax21 receptor. How can RaxH, a predicted inner membrane bound kinase with a periplasmic sensor domain, detect the Ax21 protein? Ax21 may be imported into the periplasm via a channel located in the outer membrane. For example, the *E. coli* extracellular small protein, colicin M (29 kDa), is localized to the periplasm via the FhuA porin located in the outer membrane [17]. Alternatively, Ax21 may form a structure that allows it to directly integrate into the membrane.

The observation that Ax21 is a QS factor that controls density-dependent expression of genes involved in motility, c-di-GMP turnover, and biofilm formation, suggests that PXO99*Δax21* strains would be impaired in virulence. However, earlier experiments indicated no significant changes in virulence phenotypes when PXO99*Δax21* infection was tested by clipping rice leaves with bacteria dipped in high-density cultures (10^8^ CFU/ml) [3], [18]. Because under field conditions, *Xoo* infection through hydathodes or wounded sites requires only a low inoculation density (10^4^ CFU/ml) to initiate infection [19], we hypothesized that an effect of Ax21 on virulence has been masked by the high-density inoculation approach.

To test this hypothesis, we established a new inoculation method. *Xoo* strains PXO99, PXO99Δ*raxST*, and PXO99Δ*ax21* strains were cultured in PSA (peptone sucrose media) plates and then diluted with water to 10^3^ CFU/ml. Unclipped rice leaves were then soaked in bacterial suspensions for two days, and bacterial populations assessed two days following inoculation. We found that the population of the wild-type PXO99 strain is two fold higher than that of the PXO99Δ*raxST* and PXO99Δ*ax21* strains using the low density soaking method (Figure 3D). In contrast, the populations of all three strains are similar two days after inoculation using the high-density scissor clipping method (Figure S12). These results indicate that *ax21* and *raxST* are required for full virulence during early stages of infection that mimic field conditions.

To investigate the mechanism with which Ax21 regulates motility, virulence, and biofilm formation, we generated *Xoo* strains mutated for twelve genes that are regulated by Ax21 (table S9 with the primers listed in table S10). Virulence of five strains (PXO99*Δ*01391, PXO99*Δ*01395, PXO99*Δ*02671, PXO99*Δ*04882, and PXO99*Δ*06202) is partially or completely lost in the knockout mutants. Six strains (PXO99*Δ*00678, PXO99*Δ*01395, PXO99*Δ*02637, PXO99*Δ*02671, PXO99*Δ*04882, and PXO99*Δ*06202) displayed a reduction in biofilm formation and eleven strains partially lost swimming motility (Figure S13). These analyses indicate that Ax21 exerts its complex control through regulation of target genes.

The discovery that a small protein from a Gram-negative bacterium has a dual role in QS and in activation of the host innate immune response has not previously been demonstrated. We do not, however, believe this is an anomaly or that the biological importance of Ax21 is restricted to plant pathogens. For example, we previously reported that Ax21 is also conserved in the nosocomial pathogen *Stenotrophomonas maltophilia* and proposed a similar role for Ax21 in this species [3]. Consistent with our hypothesis, a synthetic Ax21 protein has been shown to regulate gene expression, motility, and biofilm formation in *S. maltophilia,* extending our findings to an animal pathogen [20]. Furthermore, analysis of the genome sequences of other Gram-negative bacteria reveals an abundance of TOSS predicted to cleave N-terminal leader sequences and secrete mature proteins [21].

These results suggest that not only do these other Gram-negative bacteria use N-terminal processed small proteins for QS, but that some of the hundreds of the predicted receptors in rice and other species, for which no corresponding conserved microbial signature has yet been identified, detect such molecules [22]. Such knowledge can be used to develop reagents to immunize hosts against infection or antagonists to disrupt QS-mediated virulence activities and biofilm formation [23], a process thought to be involved in 65-80% of bacterial infections of plants and animals [24].

## Materials and Methods

### Bacterial strains and growth conditions

The *Xanthomonas oryzae* pv. *oryzae* (*Xoo*), *Escherichia coli* strains and plasmids used are listed in Table S11. Peptone sucrose media (PSM) [25] and nutrient broth (NB) (Difco Laboratories), containing 20 µg/ml of cephalexin (MP Biomedicals), and/or other antibiotics as appropriate were used for growing cultures of *Xoo* at 28°C. *E. coli* strains were cultured in Luria-Bertani (LB) medium at 37°C. For *E. coli,* kanamycin at 50 µg/ml, ampicillin at 100 µg/ml, cephalexin at 15 µg/ml and gentamycin at 25 µg/ml (10 µg/ml for *Xoo*) were used for selection of transformants. Rice varieties Taipei 309 (TP309, a rice line susceptible to PXO99 and a TP309 transgenic line (106-17-3-37) carrying the *Xa21* gene (TP309-XA21, resistant to *Xoo* strain PXO99) [2] were used to assess biological activity of the *Xoo* strains.

### Construction of *Xoo* knockout mutants by marker exchange mutagenesis

*Xoo* knockout mutants were generated using marker exchange mutagenesis [26]. For homologous recombination in PXO99, DNA fragments were synthesized using the polymerase chain reaction (PCR) method. Primer sequences used for each gene are shown in Table S8. PCR was carried out using Programmable Thermal Controller (MJ Research). The amplified DNA fragments were cloned into the pGEM®-T-easy vector. A kanamycin-resistant cassette was inserted into the appropriate restriction enzyme cleavage site. Sequencing of the The pGEM®-T-easy constructs carrying the mutagenized genes was performed using the dideoxy chain termination method and an automated sequencer (Model 400 I, Li-Cor) with M13 forward and reverse primers or specific primers designed based on sequencing data. Confirmed constructs were then introduced into competent PXO99 wild type cells. After electroporation, the cells were incubated for 3 h at 28°C with PS broth media, and then spread on PS agar plates containing 50 µg/ml of kanamycin. Colonies that grew on those plates were duplicated onto PS agar plates containing 50 µg/ml of kanamycin as well as plates containing 50 µg/ml of kanamycin/ampicillin in order to select for double cross-over events. Colonies that only grew on the kanamycin plates were collected and confirmed as insertional mutants using PCR. The primers that were used for gene cloning were used also used to confirm that each gene had been knocked out in these strains.

### Construction of recombinant Ax21 and generation of *Xoo* mutants expressing the recombinant protein

To generate recombinant *ax21*, a 21-bp 6x-His tag was added to the C-terminal region as follows: The *ax21* gene was amplified from the genome of PXO99 with the following primers: 5′- GTCGACGATGCAGCTCCATCCGTGTG-3′ and 5′- GTCGACTTAATGATGATGATGATGATGCCAGCTGAAGCGCGGGCCGA-3′ using the PCR method with Taq polymerase in a Programmable Thermal Controller (MJ Research Inc.). The amplified fragment was then inserted into pGem®-T Easy (Promega). The pGem®-T Easy vector containing the *ax21* gene (pGem-Ax21) was extracted and treated with the restriction enzymes *Sal*I. This fragment was then inserted into the pML122 vector [26], [27] to promote expression (pML122-rAx21) in *Xoo* and introduced into the PXO99*Δax21* [3] by electroporation. After incubation in PS broth for 3 hours, the cells were spread onto PS agar plates containing 10 µg/ml of gentamycin and 50 µg/ml of kanamycin [PXO99*Δax21*(rAx21)]. The electroporated strain was confirmed to carry the *ax21* gene by PCR using primer combinations specific for *raxST* and pML122 vector sequences. Expression of the recombinant Ax21 protein was verified by western blot analysis using a His-tag antibody and Ax21-specific antibody. For the anti-Ax21 antibody, synthetic peptides and monospecific antibodies were generated by Pacific Immunology. Detailed information about their methods can be obtained at Pacific Immunology (http://www.pacificimmunology.com/). Ax21 activity of the PXO99*Δax21*(rAx21) strain was confirmed using the scissors clipping method [3] (Figure S1).

### Purification of the recombinant Ax21 protein

The procedure for purification of recombinant Ax21 from strain PXO99*Δax21* expressing rAx21 is shown in fig. S2A. PXO99*Δax21*(rAx21) was incubated in 6 liters of nutrient broth for 3 days, harvested, and washed twice with sterilized water. The washed cells were incubated in 20 ml of modified M9 minimal media [6] for 3 days. The supernatants were collected and filtered with a 0.22 µm syringe filter to remove bacteria. Small molecules [(<7 kDa) including peptides and ions] were removed using a Zeba spin desalting column (Thermo scientific). Desalted samples were fractionated on a Superdex 75 (GE Health care) in 50 mM Na_2_HPO_4_, pH 8.0, 10 mM EDTA, 150 mM NaCl, and 0.1% Triton X-100. The flow rate of the column was set at 1 ml/min and the eluate was fractionated into 1 ml fractions. The fractions containing rAx21 were desalted again using the Zeba spin desalting column. One ml of the 50% Ni-NTA slurry was added to desalted samples and the Ni-NTA mixture incubated in 50 mM NaH_2_PO_4_, pH 8.0, 300 mM NaCl, and 10 mM imidazole for 30 minutes at room temperature. The Ni-NTA mixture was loaded onto a Poly-Prep chromatography column (BIO-RAD) and eluted with 700 µl of 50 mM Na_2_HPO_4_, pH 8.0, 300 mM NaCl containing 50, 100, 150, 200, 250, or 500 mM imidazole. All fractions were confirmed by western blot analysis using anti-Ax21 and anti-His-tag antibodies. After desalting using the Zeba spin desalting column, purified rAx21 was used for the complementation experiments.

### Silver staining

After rAx21 was purified from PXO99*Δax21*(pML122-rAx21) as described above, the fractions were separated using a 12% Sodium dodecyl sulfate polyacrylamide gel. The gel was stained with Silver stain plus (Bio-Rad) as previously described [3] (Figure S3). The fraction eluted with 150 mM imidazole buffer contained highly purified rAx21 (Figure S3, lane 6). This fraction as well as control fractions, the flow-through fraction (Figure S3, lane 3) and 250 mM imidazole buffer-eluted fraction (Figure S3 lane 8) were desalted and the used for the biological assays.

### Western blot analysis

Samples were fractionated in a 12% polyacrylamide gel. The proteins were then transferred onto Hybond ECL nitrocellulose membranes (Amersham Pharmacia Biotech) using standard procedures. The membranes were incubated with blocking solution consisting of 5% (w/v) skimmed milk in T-TBS buffer (10 mM Tris-HCl, pH 8.0, containing 150 mM NaCl and 0.1% [v/v] Tween 20) for 1 h. The membranes were then incubated in the presence of anti-Ax21 or anti-His antibody (Sigma) at a dilution of 1∶3,000 in T-TBS buffer for 1 h, and then washed with the T-TBS buffer for 10 min, three times. The membranes were then incubated for 1 h with T-TBS buffer containing a 1∶6,000 dilution of anti-rabbit IgG for anti-Ax21 and anti-mouse IgG for anti-His conjugated with horseradish peroxidase (Jackson ImmunoResearch Laboratories). After three washes with T-TBS buffer (of 15, 5, and 5 min, respectively), the membranes were incubated for 5 min with the Super Signal West Pico chemiluminescent substrate (Pierce) and then exposed to X-ray film (Fujifilm Medical Systems). Films were developed following standard autoradiographical practices.

### RNA preparation

RNA from *Xoo* PXO99 and PXO99*Δax21* harvested cells were isolated using TRIzol® reagent (Invitrogen) following the manufacturer's protocol. The RNA samples were treated with 10 units of RNase-free DNaseI (Invitrogen) for 30 min at room temperature, followed by column purification using RNeasy mini kits (Qiagen). The quality of RNA was determined by subjecting samples to gel electrophoresis on 1% agarose gels and by measuring the absorbance at 260 nm and 280 nm. Protein content in the RNA samples was assessed using A260/A280.

### cDNA generation and labeling

For Q-RT-PCR analysis, cDNA was generated by using SuperScript™III First-Strand kit (Invitrogen). One microgram of RNA was mixed with 50 ng random hexamers and 10 nMol dNTP mix. RNA mixture was incubated at 70°C for 5 min, then placed on ice for 2 min. Then cDNA synthesis mix (2 µl of 10X RT buffer, 4 µl of 25 mM MgCl_2_, 2 µl of 0.1 M DTT, 1 µl of 40U/µl RNaseOUT™, 1 µl of 200U/µl SuperScript ™III Reverse Transcriptase) was added into RNA mixture and incubated at 25°C for 10 min, followed by 50°C for 1 hour. The reactions were terminated at 85°C for 5 min, then chilled on ice. 2 U of RNase H was added and incubated at 37°C for 20 min. Synthesized cDNA was kept at −20°C until it was used as template for Q-RT-PCR analysis.

For microarray analysis, SuperScript™III Indirect cDNA Labelling System (Invitrogen) was used to synthesize label probe for microarray. Twenty microgram RNA was mixed with 3 µg random hexamers and incubated at 70°C for 5 min, then placed on ice for 2 min. Then cDNA synthesis mix (6 µl of 5X First-Strand buffer, 1.5 µl of 0.1 M DTT, 1.5 µl dNTP mix including amino-modified nucleotides, 1 µl of 40U/µl RNaseOUT™, 2 µl of 400U/µl SuperScript ™III Reverse Transcriptase) was added into RNA mixture and incubated at 25°C for 10 min, followed by 46°C for 3 hours. After cDNA synthesis, alkaline hydrolysis reaction was performed immediately to degrade the original RNA by adding 15 µl of 1 N NaOH and then incubated mixture at 70°C for 10 min. To neutralize the pH, 15 µl of 1 N HCl was mixed gently. Synthesized first strand cDNA was purified with Purification Module provided with the kit and proceeded to coupling reaction with fluorescent dye. Purified cDNA was mixed with 5 µl of 2X coupling buffer and 5 µl of DMSO in the vial of Amersham CyDye™ reactive dye (GE Healthcare Biosciences). Then labelled cDNA was purified with Purification Module and subjected to hybridization process.

### Hybridization and scanning

Labeled cDNA probes were evaporated in a vacuum centrifuge setting at 60° C to a volume of approximately 2–3 µl. Evaporated probes were then resuspended in 100 µl of a salt based hybridization solution (Ocimum Biosolutions) at room temperature. All hybridization and scanning steps were performed in a hepa and carbon filtered clean room. Hybridization was carried out using a Tecan HS 4800 hybridization station. To block nonspecific hybridization, a pre-hyridization buffer (5X SSPE, 6M Urea, 0.5% Tween-20, 10X Denhardt's solution) was applied to the slides at 50°C and agitated for 15 min on the medium setting. Labeled probes were denatured by heating the mixture at 95°C for 3 min and then cooling snapped on ice for 30 second. Probes were applied into the injector to hybridize with printed slides. Samples were hybridized for 16 hour at 42°C, then following hybridization, the slides were consecutively washed at 37°C with three salt based buffers of increasing stringency (2X SSC, 0.1% SDS, 1.0X SSC, and 0.5X SSC). Each buffer wash step was repeated twice, with a soak time of one minute followed by a one minute wash. A final wash step with water was performed. Following the final wash, slides were dried under a constant stream of N_2_ at 30°C. Slides were kept under N_2_ until scanning. Hybridized microarray slides were imaged using a GenePix 4000B dual laser microarray scanner (Axon Instruments) at 5 µm resolution. Slides were imaged using 100% laser power for both lasers (532 nm and 635 nm) and scanned twice using the high PMT and low PMT settings. All images were processed using GenePix software (Axon Instruments) for element identification and quantification. The metadata associated with the hybridizations, along with the “raw” intensities obtained from the GenePix quantitation.

### Array analysis and functional classification of differentially expressed genes

To identified differentially expressed genes from metadata, the LMGene package for R language statistic analysis that computes the p-values per gene via gene by gene ANOVA method developed by Rocke was used [28]. Genes that were differentially expressed more than 1.75 fold (log_2_ratio >0.8 or <–0.8) and have an FDR less than 5% were selected as described in our previous work [29]. To annotate the functions of the Ax21-regulated genes, COG terms (Clusters of Orthologous Groups of proteins: http://www.ncbi.nlm.nih.gov/COG/) of *Xoo* PXO99 were assigned. The TIGR Multiexperiment Viewer (MeV, http://www.tm4.org/mev.html) software was used to cluster and view expression patterns of differentially expressed genes.

### Validation of expression patterns of candidate genes using quantitative RT-PCR

To validate expression pattern from microarray analysis, the synthesized cDNA samples were diluted by adding 100 µl DEPC water. 1 µl was used as template for each reaction (10 µl). cDNA template were mixed with SYBR® Green PCR Master Mix kit (Applied Biosystems) and specific primers as listed in Table S8. Each reaction included an initial heat for 5 min at 95°C, followed by 40 cycles of PCR (95°C, 10 sec; 60°C, 20 sec). The level of gene expression of each samples were relatively calculated comparing to 16sRNA amount.

### Exogenous addition of recombinant Ax21 and quantitation of *rax* gene expression

To test whether rAx21 can restore *rax* gene expression in the PXO99*Δax21* mutant strain, we supplemented the strain exogenously with the flow-through fraction, the 150 mM imidazole-eluted fraction containing purified recombinant Ax21 (rAx21), the 250 mM imidazole buffer-eluted fraction, axY^S^22, or axM178. *Xoo* PXO99 and PXO99*Δax21* were cultured in PS broth media overnight and diluted to 10^5^ CFU/ml. rAx21, control fractions or peptides were then added exogenously and the culture continued until the cell density reached 10^8^ CFU/ml. Cultured cells were harvested and RNA isolated as described above (see RNA isolation and cDNA generation methods). The final concentration of exogenous addition to the bacterial culture was 1 µM for axY^S^22, and 5 nM for rAx21. All experiments were carried out with at least three biological replicates including four technical replicates in each experiment. All biological replicates gave similar results.

### Swimming motility assays

The impact of Ax21 regulation on bacteria swimming motility was evaluated as described previously [30]. All tested *Xoo* strains were cultured in PSB media until cell densities reached to 10^8^ CFU/ml. Cells were pelleted, washed with sterilized water twice, and resuspended to 10^9^ CFU/ml. Then 3 µl of concentrated cultures were dropped in the middle of swimming assay plate (modified minimal media containing 0.15% agar), and incubated at 28°C for three days. The diameters of expanding colonies were measured and mean values were calculated from four biological replicates.

### Virulence assays

In this study, two inoculation methods, the standard clipping [18] and the soaking method, were used for evaluation of virulence of the *Xoo* strains. For the standard clipping method, *Xoo* strains were cultured in PSB media until cell densities reached 5×10^8^ CFU/ml. Six week-old rice cultivar TP309 (susceptible to PXO99 strain) was inoculated by clipping the leaf tip with scissor that dipped into bacterial culture. The leaf lesion lengths were measured two weeks after inoculation using our standard procedures [2]. For the soaking method, rice leaves were soaked for two days in *Xoo* cultures of 10^3^ CFU/ml. Bacterial populations were determined as previously described [31] at two days after inoculation.

### Biofilm formation assays

To quantitate biofilm formation in *Xoo*, we used the polyvinyl chloride microplate method [32]. *Xoo* strains were cultured in PS broth media overnight and then diluted to concentration 5×10^5^ CFU/ml in minimal media. For complementation experiments, we supplemented the PXO99*Δax21* mutant strain exogenously with the flow-through fraction, the 150 mM imidazole-eluted fraction containing purified recombinant Ax21 (rAx21), or the 250 mM imidazole buffer-eluted fraction and then continued cultured for seven days. After seven days, the cultures remaining in the plate were removed with pipettes. The remaining cells were stained with a 0.1% crystal violet solution for 30 min and excess dye was washed twice with distilled water. Dye that stained on the adhesive cells was resuspended with 95% EtOH, the optical density was measured at 590 nm and average values from four biological replicates were calculated. The final concentration of exogenous addition to the bacterial culture is 5 nM for rAx21.

### Confocal microscopy

PXO99 and PXO99*Δax21* strains carrying a green fluorescent protein (GFP) (Han et al., 2008) were cultured in M9 minimal media with glass slides (10^5^ CFU/ml). After 4 days incubation, the glass slides with attached cells were washed nine times with sterilized water, and then air-dried. Biofilm formation was observed with a Leica True Confocal Scanner (TCS) SPE confocal microscope. The GFP was imaged under the following conditions: excitation: 488 nm; dichroic mirror: 405/488/543; emission: 495–530 nm. Images were analyzed using the program ImageJA (Ver 1.45b). After imaging, the attached bacterial cells were immediately recovered from the glass slide with 2 ml of sterilized water by extensively pipetting. The population of the recovered cells was determined using a colony counting method on PSA plates.

### Aggregation assays

PXO99 and PXO99*Δax21* strains carrying the green fluorescent protein were generated as described previously [31]. *Xoo* strains were grown on PSA plates, harvested, and washed with sterilized distilled water. The washed cells were resuspended to 10^6^ CFU/ml. The diluted cells were dropped into an 8-chamber slide and incubated for three days at room temperature. Aggregated cells were observed using a Zeiss Axiophot fluorescence microscope (Jena) equipped with a fluorescein isothiocyanate filter (excitation filter, 450 to 490 nm; emission filter, 520 nm; dichroic mirror, 510 nm).

## Supporting Information

Figure S1 Recombinant Ax21 protein is biologically active. After culturing PXO99 (blue), PXO99*ΔraxST* (red), PXO99*Δax21* (yellow), or PXO99*Δax21*(rAx21) (purple) strains on PS agar plates containing cephalexin, kanamycin, and/or gentamycin, the cells were diluted to 5×10^8^ CFU/ml and inoculated onto TP309 rice leaves (lacking XA21) and TP309-XA21 (carrying XA21) by the scissor clipping method. Each bar represents the average ± standard deviation (SD) of six sampled leaves per treatment. The experiment was repeated two times.
(TIF)

Figure S2 Silver staining and western blot analyses reveal that recombinant Ax21 is highly purified. (A) Scheme for the purification of recombinant Ax21 (rAx21). rAx21 was purified from supernatants from the PXO99Δ*ax21*(rAx21) strain using Superdex 75 for a gel filtration and an Ni-NTA for his-tag purification. Samples were run in an 12% acrylamide gel (B) Silver staining and (C) Western blot analysis using anti-Ax21 antibody. Lanes are designated as follows: M, Marker; 1, Desalted total supernatants; 2, after gel filtration chromatography; 3, flow through; 4, elution with 50 mM imidazole buffer; 5, 100 mM imidazole buffer; 6, 150 mM imidazole buffer; 7, 200 mM imidazole buffer; 8, 250 mM imidazole buffer; 9, 500 mM imidazole buffer. The arrow indicates the rAx21 protein. A band corresponding the full-length N-terminal processed rAx21 reacted with the anti-His tag antibody indicating that the mature protein is secreted.
(TIF)

Figure S3 The mature, processed rAx21 lacking the N-terminal signal peptide is secreted into supernatants. Desalted supernatants from the PXO99Δ*ax21*(rAx21) strain were digested by trypsin, and LC-MS/MS analysis carried out as described previously [2]. (A) Deduced amino acid sequence of rAx21. Yellow indicates amino acid sequence from the nine unique peptides obtained from LC-MS/MS analysis (B to J). The red box designates the predicted N-terminal signal peptide. The spectra of the nine peptides, which covered nearly the entire region of rAx21 except for the predicted N-terminal signal peptide, obtained from LC-MS/MS analysis are as follows: (B) AENLSYNFVEGDYVR, (C) TPTDGRDADGWGVK, (D) ASYAVAPNFHVFGEYSK, (E) NTNSDFQQWGVGVGFNHEIATSTDFVAR, (F) RLDLDSPNINFDGYSVEAGLR, (G) NAFGEHFEVYALAGYEDYSK, (H) GIDAGNDFYGR, (I) MDGDGNKEWSVGPR, and (J) FSWHHHHHH (include the 6x His tag).
(TIF)

Figure S4 The AxY^S^22 peptide is stable and biologically active after two days incubation with *Xoo*. Two µM of AxYS22 were incubated in (1) water, (2) PXO99, and (3) PXO99Δ*raxST* for 2 days and then supernatants were collected. As a control, supernatants from (4) PXO99Δ*raxST* culture without AxY^S^22 peptide were included. These samples were used to pretreat TP309-XA21 rice leaves as described previously [2]. After pretreatment, the rice leaves were inoculated with PXO99Δ*raxST*. Lesion lengths were measured two weeks after PXO99Δ*raxST* inoculation. Each bar indicates the average lesion length ± SD from 5 or 7 leaves.
(TIF)

Figure S5 The axY^S^22 and axM178 peptides derived from the Ax21 protein do not confer QS activity. Expression of the *raxST* (left), *raxB* (middle), and *raxR* (right) genes from PXO99 at 10^8^ CFU/ml, PXO99 at 10^6^ CFU/ml, and PXO99 at 10^6^ CFU/ml supplemented with (A) axY^S^22 or (B) axM178 peptides, which were previously identified in biologically active fractions [3], was assessed using Q-RT-PCR with primers specific to each gene. Primers are as listed in table S8. Levels of gene expression were calculated relative to 16sRNA expression. Data are the mean of three replicates ± standard deviation (SD).
(TIF)

Figure S6 Lack of the *Xoo raxST* significantly reduces Ax21-mediated QS. Density dependent expression of the genes from PXO99 at 10^8^ CFU/ml, PXO99 at 10^6^ CFU/ml, and PXO99 at 10^6^ CFU/ml with exogenous addition of rAx21 isolated from 1, PXO99*Δax21*(rAx21) or 2, PXO99*ΔraxST* was assessed as described in Materials and Methods. Levels of gene expression were calculated relative to 16sRNA expression. Primers specific to *raxST* are as listed in table S8. Data are the mean of three replicates ± standard deviation (SD).
(TIF)

Figure S7 Expression of ten Ax21 regulated genes is validated by Q-RT-PCR analysis. To validate the microarray results, we assessed expression levels of ten Ax21-regulated genes (from the 10^8^ CFU/ml dataset) using Q-RT- PCR with specific primers as listed in Table S8. The relative fold change of transcriptional levels in PXO99 and PXO99*Δax21* strains were determined by microarray analysis (grey) and Q-RT-PCR (black) (+  =  expression level of PXO99 is higher than of PXO99*Δax21*, -  =  expression level of PXO99 is lower than of PXO99*Δax21*). Although the amplitude of the observed gene expression fold changes differ between the two techniques, as might be expected due to their sensitivity, the general trend of gene expression is similar.
(TIF)

Figure S8 COG enrichment analysis indicates that Ax21 controls density-dependent expression of genes controlling diverse bacterial processes. To predict putative biological functions of Ax21 we applied COG (Cluster of Orthologous Groups of proteins) enrichment analysis. Each Ax21-regulated gene was assigned a COG term and grouped according to its biological function (http://www.ncbi.nlm.nih.gov/COG/). The numbers of Ax21-regulated genes in each functional category were calculated as a percentage of the total number of Ax21-regulated genes in each dataset (early log, mid log, and late log). Then the percentage of Ax21-regulated genes of each functional category was divided by the original percentage of each functional category present in the array platform (total numbers of genes in one functional categories/total numbers of genes on the array platform). The ratios between percentage of Ax21-regulated gene number and arrays in each category are presented in a pseudocolor numeric scale (Yellow, Ax21 up-regulated; Blue, Ax21 down-regulated). This analysis indicates that when cell population density is low, Ax21 controls up-regulation of genes (red box) involved in cell motility, cell cycle, inorganic ion metabolism, defense mechanism, coenzyme metabolism, and intracellular trafficking, but down-regulation of genes (green box) involved in transcription and translation. In contrast, when cell population density is high, Ax21 up-regulates genes (green box) involved in transcription and translation. The pattern of COG enrichment, created by MeV (www.tm4.org/mev, Multi experiment Viewer), of the microarray data supports our finding that Ax21 is a quorum sensing factor that controls diverse gene functions.
(TIF)

Figure S9 Whole genome transcriptomics of PXO99 vs. PXO99*Δax21* at three different population densities. (A) A heat map represents the ratio of gene expression levels in a log_2_-based pseudocolor scale in (i) late log phase (10^8^ CFU/ml), (ii) early log phase (10^6^ CFU/ml) (red, Ax21-up-regulated; green, Ax21-down-regulated). (B) Expression profiles of selected Ax21-regulated genes that are highly expressed at high population densities reveal an enrichment for putative transcriptional regulators. Of these, only the *colR* response regulator has been characterized (up-regulated 2 fold in PXO99 vs. PXO99Δ*ax21*). *colR* is critical for host colonization and infection in *P. flurorescens* and *X. campestris* pv. *campestris,* respectively. Our analysis also revealed that a gene encoding a (ppGpp)ase (ppGpp, guanosine-3,5-bispyrophosphate) is up-regulated by Ax21 suggesting that Ax21 controls ppGpp turnover.
(TIF)

Figure S10 PXO99Δ*ax21* shows significantly reduced biofilm formation compared with PXO99. (A) Biofilm formation assay on glass slides was performed using PXO99 and PXO99Δ*ax21* strains carrying a green fluorescent protein as described in Materials and Methods. GFP was imaged under the following conditions: excitation: 488 nm; dichroic mirror: 405/488/543; emission: 495–530 nm. Width (X) x Height (Y) x Depth (Z): 1.1 × 1.1 × 0.141 mm. (B) Images were analyzed using the program ImageJA (Ver 1.45b). After imaging, the attached bacterial cells were immediately recovered from the glass slides with 2 ml of sterilized water by extensively pipetting. The population of the recovered cells was determined using a colony counting method. Bars indicate average of three replicates ±SD.
(TIF)

Figure S11 PXO99Δ*raxH* does not respond to exogenous addition of Ax21. PXO99, PXO99Δ*phoQ*, PXO99Δ*raxH*, and PXO99Δ*ax21* strains (5×10^5^ CFU/ml), with or without purified rAx21, were tested for biofilm formation as described in Materials and Methods. The higher OD reflects more biofilms formed. Bars indicate average of four biological replicates ±SD.
(TIF)

Figure S12 Growth of PX099, PXO99Δ*raxST* and PXO99Δ*ax21* strains using the scissors clipping method. TP309 rice leaves were inoculated by clipping the leaf tip with scissors dipped into *Xoo* cultures of 5×10^8^ CFU/ml. PXO99, PXO99Δ*raxST,* and PXO99Δ*ax21* strains were extracted from rice leaves two days after inoculation and populations quantified using established procedures [3]. Each bar indicates the average of nine leaves ± SD. Four replicate experiments gave similar results.
(TIF)

Figure S13 Phenotypic validation of twelve selected Ax21-regulated genes. Twelve of the Ax21-regulated genes listed in Table S9 were selected for knockout analysis using the marker exchange mutagenesis method (primers listed in Table S10). All *Xoo* mutant strains, generated in this study, were tested for (A) Swimming motility, (B) virulence (by standard clipping method), and (C) biofilm formation. Each bar represents the average ± standard deviation (SD). Mutations in genes that are regulated by Ax21 show phenotypic defects in the PXO99*Δax21* strain compared to PXO99. These results indicate Ax21 controls the observed phenotypes through regulation of the Ax21-regulated genes. Nine of the twelve gene tested have been previously characterized in *Xanthomonas spp* or other bacteria. Three genes encode hypothetical proteins containing putative GGDEF and EAL domains. Strains carrying knockouts in these three genes also displayed reduced biofilm, swimming motility and virulence phenotypes.
(TIF)

Table S1 Density-dependent expression of *rax* genes is controlled by Ax21.
(DOCX)

Table S2 Genes up-regulated in early log phase by Ax21.
(DOCX)

Table S3 Genes up-regulated in mid log phase by Ax21.
(DOCX)

Table S4 Genes up-regulated in late log phase by Ax21.
(DOCX)

Table S5 Genes down-regulated in early log phase by Ax21.
(DOCX)

Table S6 Genes down-regulated in mid log phase by Ax21.
(DOCX)

Table S7 Genes down-regulated in late log phase by Ax21.
(DOCX)

Table S8 List of primers used for quantitative realtime PCR.
(DOCX)

Table S9 Expression profile of *Xoo* genes that were selected to generate knockout strains for functional analysis.
(DOCX)

Table S10 List of primers used to generate *Xoo* knockout strains.
(DOCX)

Table S11 Bacterial strains and plasmids used in this study.
(DOCX)
